This article has been retracted.

# Identification of *MMP9* as a Novel Biomarker to Mitochondrial Metabolism Disorder and Oxidative Stress in Calcific Aortic Valve Stenosis

**DOI:** 10.1155/2022/3858871

**Published:** 2022-09-24

**Authors:** Cong Liu, Ruixue Liu, Zhezhe Cao, Qiao Guo, He Huang, Liangming Liu, Yingbin Xiao, Chenyang Duan, Ruiyan Ma

**Affiliations:** ^1^Department of Cardiovascular Surgery, Xinqiao Hospital, Army Medical University, Chongqing 400037, China; ^2^Department of Ultrasound Medicine, Union Hospital, Tongji Medical College, Huazhong University of Science and Technology, Wuhan 430022, China; ^3^Department of Anesthesiology, The Second Affiliated Hospital of Chongqing Medical University, Chongqing 400010, China; ^4^Department of Shock and Transfusion, State Key Laboratory of Trauma, Burns and Combined Injury, Daping Hospital, Army Medical University, Chongqing 400042, China

## Abstract

Calcific aortic valve stenosis (CAVS) is the most common heart valve disorder among humans. To date, no effective method has been identified to prevent this disease. Herein, we aimed to identify novel diagnostic and mitochondria-related biomarkers of CAVS, based on two machine learning algorithms. We further explored their association with infiltrating immune cells and studied their potential function in CAVS. The GSE12644, GSE51472, and GSE83453 expression profiles were downloaded from the Gene Expression Omnibus (GEO) repository. The GSE12644 and GSE51472 datasets were integrated to identify differentially expressed genes (DEGs). GSE12644 contains 10 normal and 10 CAVS samples, whereas GSE51472 contains 5 normal and 10 CAVS samples. GO and KEGG assays of DEGs were conducted, and the correlation between matrix metalloproteinase 9 (*MMP9*) expression and immune cell infiltration was explored, using CIBERSORT. The LASSO regression model and SVM-RFE analysis were used to identify diagnostic genes. The expression of *MMP9* in CAVS and non-CAVS samples was measured using RT-PCR, western blotting and immunohistochemistry. A series of functional experiments were performed to explore the potential role of *MMP9* in mitochondrial metabolism and oxidative stress during CAVS progression. Twenty-two DEGs were identified, of which six genes (*SCG2*, *PPBP*, *TREM1*, *CCL19*, *WIF1*, and *MMP9*) were ultimately distinguished as diagnostic genes in CAVS. Of these, *MMP9* was indicated as a mitochondria-related gene, the expression and diagnostic value of which were further confirmed in the GSE83453 dataset. Correlation analysis revealed a positive correlation between *MMP9* and infiltrating immune cells. In our cohort, *MMP9* expression was distinctly increased in CAVS samples, and its inhibition attenuated the calcification of valve interstitial cells (VICs) by suppressing mitochondrial damage and oxidative stress. Taken together, our findings suggest *MMP9* as a novel mitochondrial dysfunction biomarker and therapeutic target for CAVS.

## 1. Introduction

Valvular heart disease (VHD) comprises a wide range of common cardiovascular disorders, accounting for 10 to 20% of all cardiac surgical procedures in the United States [1]. Calcific aortic valve stenosis (CAVS) is widely regarded as the most common form of VHD. It is also a predominant cause of aortic valve stenosis [2], worldwide. Surgical or transcatheter valve replacement is inevitable in the absence of a pharmacological cure for this common and progressive condition. As the most common heart valve condition in developed countries, aortic stenosis affects approximately 3% of the population aged over 65. The survival rates of asymptomatic patients with aortic stenosis are comparable to those of age- and sex-matched control cases [3]. However, the long-term survival in symptomatic cases without aortic valve replacement is merely 2 to 3 years [4]. Aortic valve calcification remains a mystery despite advancements in drastic therapies, such as valve replacement, and established interventional therapies for treating aortic stenosis. Therefore, it is critical to study the progression of CAVS and identify the molecules that are essential to its development, to facilitate timely identification and treatment of patients.

Mitochondria, the main organelles of aerobic respiration, are of great significance for maintaining the normal physiological function of cells [5, 6]. Under normal conditions, the mitochondrial quality indices—including mitochondrial dynamics, functions, and metabolism—are in dynamic balance [7]. Our previous study [2] confirmed the existence of a severe mitochondrial quality imbalance in calcified valves, which mainly manifests as mitochondrial morphological damage. This includes mitochondrial fragmentation, mitochondrial dysfunction (such as excessive ROS accumulation), reduction of mitochondrial membrane potential, and mitochondrial metabolic disorders, such as the obvious downregulation of glutathione metabolism and the tricarboxylic acid (TCA) cycle. The study of Tandon et al. [8] showed that changes in mitochondrial morphology may lead to the accumulation of collagen matrix in valve interstitial cells (VICs), which can be used as an index to evaluate early CAVS. The study of Morciano et al. [9] showed that mitochondrial dysfunction can promote the synthesis of collagen matrix and alkaline phosphatase of VICs and accelerate the calcification process of CAVS. The study of Khatun et al. [10] indicated that the disorder of mitochondrial metabolism may accelerate the synthesis of alkaline phosphatase and the osteogenic-like changes of VICs. The above researches fully confirmed that the mitochondrial quality imbalance in VICs has important regulatory significance for the occurrence and development of CAVS. Therefore, it is essential to identify an effective mitochondrial marker for severity prediction of CAVS.

In recent years, microarray technology—together with comprehensive assays—has been used to identify new functional genes related to a variety of disorders [11, 12]. These genes could be used as possible markers for the diagnosis and prognosis of various diseases. In the past decade, a growing number of studies have used machine learning algorithms to screen diagnostic genes and potential functional factors of various diseases. However, the application of such machine learning algorithms for screening novel biomarkers for CAVS has rarely been reported.

In this study, we obtained two public microarray datasets (GSE12644 and GSE51472) on CAVS from the Gene Expression Omnibus (GEO) database and screened for differentially expressed genes (DEGs) between CAVS and non-CAVS samples. Moreover, we used machine learning algorithms to identify potential diagnostic mitochondrial genes for CAVS and further performed a series of experiments to confirm our findings.

## 2. Materials and Methods

### 2.1. Clinical Samples

Calcified valve specimens were obtained from 15 patients with CAVS (CAVS group) who had undergone surgical treatment at the Xinqiao Hospital of the Army Medical University (Chongqing, China). Valve samples for the non-CAVS group were obtained from 15 patients with aortic insufficiency but no calcification. This study was approved by the Ethics Committee of the Institute of Biomedicine Research of Xinqiao Hospital of the Army Medical University (No. 2022-YAN187-01).

### 2.2. Cell Culture and Calcification

Noncalcified aortic valves were used for the isolation of human aortic valve interstitial cells (VICs). Primary VICs were isolated, and the quality of the cell preparation was verified in the control media (CM). Osteogenic differentiation was induced in cells from passages 3 to 7 by incubating cells with osteogenic medium (OM) for 28 days. The osteogenic medium included 0.1% fetal bovine serum, 50 *μ*g/ml ascorbic acid, and 5 mmol/l *β*-glycerol phosphate (all purchased from Sigma-Aldrich, St. Louis, MO, USA). The medium was changed every 4 days, as previously described [13].

As for inhibiting matrix metalloproteinase 9 (*MMP9*) expression in OM-VICs, the primary VICs were treated with MMP-9-IN-1 (MMP-9i) accompanied by osteogenic differentiation treatment at a concentration of 100 or 300 nM. MMP-9i was a *MMP9*-specific inhibitor which was purchased from Selleck (Shanghai, China) [14].

### 2.3. Alizarin Red Detection

The VICs were then fixed in 10% neutral formaldehyde at room temperature for 30 minutes, after the removal of the calcification medium, and washed two to three times with ultrapure water. 3 ml of 0.5% Alizarin Red staining solution (Beyotime, Shanghai, China) was added, and the plate gently shaken on a shaking table for 5–10 minutes, to allow dyeing. Excess dye was removed by pipette suction, and 1 ml ultrapure water was added to each well of the six-well plate. The mixture was shaken for a further 5 minutes before being washed with ultrapure water for four iterations of 5 minutes each. Finally, the preparation was washed with phosphate-buffered saline (PBS) for 15 minutes, excess PBS was absorbed, and the ultrapure water was added to the wells, prior to photography and quantification.

### 2.4. Real-Time PCR

TRIzol reagent (Invitrogen, Carlsbad, CA, USA) was used to extract total RNA from the specimens, according to the manufacturer's instructions. Reverse transcription was executed using HiScript II RT SuperMix for qPCR (+gDNA wiper) (Vazyme Biotech, Nanjing, China) and 1 ng RNA. SYBR Green Master Mix (Vazyme Biotech) was used to conduct real-time PCR according to the following parameters: the reaction mixture was heated to 95°C for 2 minutes, followed by 34 cycles of 94°C denaturation for 50 seconds, annealing for 45 seconds, and 72°C extension for 50 seconds. Glyceraldehyde 3-phosphate dehydrogenase (GAPDH) was used as an internal reference to standardize the expression data. The primer sequences of human MMP-9 and GAPDH were shown as follows: MMP9_forward: CGTGAACATCTTCGACGCCAT, reverse: CGCTCCTCAAAGACCGAGTCCA, GAPDH_ forward: CAACAGCCTCAAGATCATCAGCA, reverse: ATGAGTCCTTCCACGATACCAA. The relative expression was determined using the following equation:

(1) $$\begin{array}{c} 2-\Delta \Delta Ct\;\left(\Delta Ct=\Delta Cttar–et-\Delta CtGAPDH\right). \end{array}$$

### 2.5. Western Blotting

Aortic valve tissue was preserved at -80°C. Sodium dodecyl sulfate-polyacrylamide gel electrophoresis (SDS-PAGE) was used to separate the total protein in a lysis solution, followed by electroblotting to transfer the protein onto polyvinylidene fluoride membranes. Antibodies were incubated on the membrane, overnight at 4°C, after being blocked with the Odyssey blocking buffer (LI-COR, Shanghai, China). Subsequently, the membranes were incubated with a horseradish peroxidase-conjugated secondary antibody, for 1 hour. GAPDH was used as an endogenous control. Mouse anti-human GAPDH polyclonal antibody (1 : 5000, Abcam, Cambridge, MA, USA) was used to detect GAPDH. The protein level of *MMP9* was examined using a mouse anti-human *MMP9* polyclonal antibody (1 : 3000, Abcam, Cambridge, MA, USA). Proteins were detected using ECL Plus kits (Thermo Scientific, Waltham, MA, USA), and Image-Pro Plus Version 6.0 was used for analysis.

### 2.6. Immunohistochemistry

For semiquantitative examination, tissue samples were fixed with 10% formalin at room temperature for 24 hours, embedded in paraffin, and cut into 20 *μ*m-thick sections. Immunohistochemical staining for *MMP9* was also performed. Briefly, sections were washed and blocked using 5% milk in Tris-buffered saline, at room temperature for 2 hours. Primary antibodies were incubated overnight with the tissue slices, at 4°C. The sections were then washed in PBS and incubated for 30 minutes with biotinylated secondary antibodies, prior to treatment with VECTASTAIN ABC reagent (Vector Laboratories, Inc., Burlingame, CA, USA) and 3,3′-diaminobenzidine (Sigma-Aldrich, St. Louis, MO, USA), for 2 minutes at room temperature, followed by counterstaining with hematoxylin. Images were captured using an optical microscope without any filters. Signal quantification was performed using the Image-Pro Plus software.

### 2.7. Mitochondrial Morphology Detection

Mitochondria in VICs were labeled using 100 nmol/l MitoTracker Deep Red (Thermo Fisher Scientific, Waltham, MA, USA) at 37°C for 30 minutes, and observed using confocal microscopy (Leica TCS SP5, Wetzlar, Germany), using a ×60, 1.3 NA oil-immersion objective. Mitochondrial fluorophores were excited using a 633 nm laser, and fluorescence emission was recorded at 558–617 nm. Mitochondrial length was determined and calculated using the ImageJ software.

### 2.8. FITC-ROS Assay

VICs were stained with 1% DCFH-DA or dihydroethidium (DHE) fluorescent probes, incubated at 37°C for 20 min, and observed using confocal microscopy (Leica TCS SP5, Wetzlar, Germany), using a ×40 objective as well as differential and interference contrast (DIC). The ROS fluorescence was excited by a 488 nm laser and emission was collected at 501–563 nm. Quantification for the ROS assay was conducted using ImageJ to measure the FITC fluorescence intensity [5, 6].

### 2.9. Mitochondrial Membrane Potential Assay

VICs were stained with 0.1% JC-1 fluorescent probes and incubated at 37°C for 20 min. The JC-1 monomer was excited by a 488 nm laser, and emission was collected at 500-650 nm. The JC-1 aggregate fluorescence was excited by a 633 nm laser and emission was collected at 558-617 nm. Quantification for mitochondrial membrane potential was carried out to measure the fluorescence intensity ratio of JC-1 aggregate/JC-1 monomer [5, 6].

### 2.10. Microarray Data

We retrieved the gene expression profiles, GSE12644 and GSE51472, from the GEO database. These datasets included the expression data of aortic valves—from patients with CAVS, as well as normal controls—which were detected on the GPL570 platform. GSE12644 contains 10 normal and 10 CAVS samples from Canada, whereas GSE51472 contains 5 normal and 10 CAVS samples. In addition, the GSE83453 dataset, which includes 8 normal tricuspid valves, 9 stenotic tricuspid valves, and 10 calcified bicuspid aortic valves, was used as the validation cohort.

### 2.11. DEG Analysis

The data table of the microarray platform was used to annotate the two series matrix files (GSE51472 and GSE12644) with official gene symbols, whereafter gene expression matrix files were obtained. The two datasets were merged into one file, and the “sva” R package was applied to perform batch normalization of the expression data. The DEG analysis was conducted using the “limma” R program. The threshold for DEGs was set as |log2(*fold* − *change*)| > 1 and *p* < 0.05.

### 2.12. Enrichment Analysis of DEGs

As a predominant bioinformatics tool for the annotation of genes, Gene Ontology (GO) analysis describes three categories of gene functions, namely, biological process (BP), molecular function (MF), and cellular component (CC). Information regarding genomes, biological pathways, diseases, and chemicals were derived from the Kyoto Encyclopedia of Genes and Genomes (KEGG). The clusterProfiler package was applied in RStudio 1.1.456 (RStudio, Boston, MA, USA) to perform GO functional enrichment analysis and KEGG pathway assays on the DEGs.

### 2.13. LASSO Model and SVM-RFE Methods

The diagnostic indicators of CAVS were classified using LASSO logistic regression and the support vector machine (SVM) algorithm. LASSO analysis was conducted using the “glmnet” package, for which the response type was set to binomial and the alpha, to 1. Both classification and regression may benefit from using an SVM. A recursive feature elimination (RFE) method was used to select the best genes from the meta-data cohort, to avoid overfitting. Therefore, support vector machine-recursive feature elimination (SVM-RFE) was used to discover the set of genes with the greatest discriminative ability. A total of 1513 mitochondria-related genes were identified via gene set enrichment analysis.

### 2.14. Comprehensive Correlation Analysis of Infiltrating Immune Cells

Based on normalized gene expression patterns, CIBERSORT can be used to measure infiltrating immune cell fractions [15]. To estimate the abundance of distinct immune cell types in the immunological microenvironment, CIBERSORT employed TPM data from RNA-seq, which were transformed from FPKM data. A total of 100 aligned, default signature matrices were obtained from the CIBERSORT website (https://cibersort.stanford.edu/index.php) to conduct gene expression analysis. A correlation analysis in R was performed to examine the relationship between new genes and quantities of invading immune cells. Results were displayed in the form of a chart, constructed using the “ggplot2” program.

### 2.15. Statistical Analysis

All statistical analyses were conducted using R (version 3.6.3) and SPSS 17.0 for Windows (SPSS Inc., Chicago, IL, USA). Comparisons between two independent groups were analyzed using Student's *t*-test. Statistical significance was set at *p* < 0.05.

## 3. Results

### 3.1. Identification of DEGs in CAVS and Functional Enrichment Analysis

Following GSE12644 and GSE51472 dataset analysis, 22 DEGs were identified, which included 4 downregulated and 18 upregulated genes (Figure 1(a)). The KEGG pathway enrichment and GO annotation analysis using clusterProfiler were conducted to gain a better understanding of the biological roles played by the identified DEGs. The GO and KEGG pathways are shown in Figures 1(b) and 1(c), respectively. BP assays indicated that 22 DEGs were mainly enriched in “extracellular matrix organization,” “extracellular structure organization,” “external encapsulating structure organization,” and “ossification.” For CC assays, the top four distinctly enriched terms were “collagen-containing extracellular matrix,” “endoplasmic reticulum lumen,” “tertiary granule,” and “secretory granule lumen.” The top four distinctly enriched MF terms included “cytokine activity,” “receptor ligand activity,” “signaling receptor activator activity,” and “G protein-coupled receptor binding” (Figure 1(b)). In addition, the data from KEGG assays confirmed that the 22 DEGs were mainly enriched in the “IL-17 signaling pathway,” “ECM-receptor interaction,” “viral protein interaction with cytokine and cytokine receptor,” “chemokine signaling pathway,” and “focal adhesion” (Figure 1(c)).

### 3.2. Identification of Diagnostic Genes Using Two Machine Learning Algorithms

We used two alternative methods to identify biomarkers. CAVS diagnostic biomarkers were reduced using LASSO regression analysis, which resulted in the identification of six genes (Figure 2(a)), whereas nineteen of the twenty-two DEGs were screened using the SVM-RFE algorithm (Figure 2(b)). Six overlapping genes (*SCG2*, *PPBP*, *TREM1*, *CCL19*, *WIF1*, and *MMP9*) were ultimately identified between the two machine learning algorithms (Figure 2(c)). To further identify whether any mitochondria-related genes resided among these six biomarkers, we constructed a Venn diagram and found that *MMP*9 met the relevant conditions (Figure 2(d)). Therefore, we focused on *MMP9* expression in this study. We proceeded to analyze the GSE83453 dataset, which also confirmed that *MMP9* expression was distinctly upregulated in CAVS samples compared with normal samples (Figure 3(a)). Moreover, the receiver operating characteristic (ROC) curve analysis revealed that *MMP9* was a potential indicator to distinguish CAVS samples from normal samples, with an area under the curve (AUC) of 0.921 (95% CI, 0.743–0.1000, *p* < 0.001; Figure 3(b)). Furthermore, the results of ROC assays on GSE12644 and GSE51472 exhibited similar results (Figure 3(c)).

### 3.3. Relationships between the Expression of *MMP9* and Infiltrating Immune Cells

The function assays discussed above revealed that the “chemokine signaling pathway,” “viral protein interaction with cytokine and cytokine receptor,” “ECM-receptor interaction,” “IL-17 signaling pathway,” and “focal adhesion” were noticeably enriched. Therefore, we questioned whether *MMP9*'s harmful impact in CAVS was mediated through immune cell infiltration. Accordingly, we used CIBERSORT techniques to investigate the relationship between *MMP9* expression and invading immune cells, in CAVS. Twenty-two types of immune cell profiles identified from CAVS and normal samples are shown in Figures 4(a) and 4(b). In addition, we found that the levels of M2 macrophages were distinctly decreased in CAVS samples compared with those in normal samples (Figure 4(c)). The results of the correlation analysis showed that *MMP9* was positively correlated with “macrophage M0,” “dendritic cells activated,” and “macrophage M2” (Figures 5(a) and 5(b)). Our findings suggested that *MMP9* expression is substantially correlated with immune cell infiltration in CAVS.

### 3.4. Distinct Upregulation of *MMP9* and Its Potential Role in Mitochondrial Metabolism and Oxidative Stress in CAVS Progression

To determine whether a dysregulated level of *MMP9* was exhibited in CAVS, we collected 15 CAVS and non-CAVS samples, respectively. RT-PCR and western blotting experiments revealed that the expression of *MMP9* was distinctly upregulated in CAVS samples, compared to that in non-CAVS samples (Figures 6(a) and 6(b)). A similar result was also observed using immunohistochemistry (Figure 6(c)). The computed tomography (CT) imaging confirmed the presence of a significantly calcified focus in the CAVS samples. At the same time, we found that the mitochondria in CAVS samples were seriously damaged, with severe vacuolation of the internal cristae (Figure 6(d)). To further explore the possible roles of *MMP9* dysregulation in mitochondrial function, we performed precalcification in VICs with osteogenic medium (OM) and found that the mitochondria were significantly fragmented, confirming the existence of mitochondrial damage in calcified VICs. *MMP9* inhibition by MMP-9i (Figure S1) could significantly improve mitochondrial morphology in calcified VICs (Figure 7(a)). The fluorescence intensity of FITC-ROS DCFH-DA (Figure 7(b) and S2) and DHE (Figure 7(c)) was significantly increased, indicating that the oxidative stress occurred in calcified VICs. The fluorescence intensity ratio of JC-1 aggregate/JC-1 monomer was markedly decreased (Figure 7(d) and S3), suggesting that the mitochondrial membrane potential reduced in calcified VICs. *MMP9* inhibition by MMP-9i could significantly attenuate mitochondrial dysfunctions (Figures 7(b)–7(d)). Besides, the citrate synthase activity was markedly reduced in calcified VICs (Figure 7(e)), indicating the existence of mitochondrial metabolism disorder in calcified VICs. *MMP9* inhibition by MMP-9i could also enhance the citrate synthase activity of VICs. The above results suggested that inhibiting *MMP-9* may attenuate the mitochondrial quality imbalance of calcified VICs in a dose-dependent manner. In addition, the calcification of VICs was also decreased significantly in a dose-dependent manner (Figures 7(a)–7(e)). Overall, our findings suggested that *MMP9* is highly expressed in CAVS and plays a critical role in the mitochondrial quality imbalance observed in calcified VICs.

## 4. Discussion

According to our current understanding, CAVS is a dynamic condition characterized by lipid accumulation, persistent inflammation, and active valve leaflet calcification [16]. Valvular degeneration precedes aortic stenosis and is characterized by calcification of the aortic valves, which is initially mild or moderate before worsening, with or without clinical symptoms [17]. CAVS progresses over a lengthy period and its presentation varies greatly from person to person. To date, potential prognostic biomarkers for CAVS have been limited. In recent years, an increasing number of studies have used machine learning techniques to screen novel biomarkers for various diseases, including those of the cardiovascular system [18, 19]. The artificial intelligence subfield of machine learning makes use of massive datasets to create predictions. Although most algorithms used in machine learning had been developed as far back as the 1950s, this technology has been resurrected over the past two decades [20], owing to the rise of big data and improved computational power.

In our study, we screened DEGs between CAVS and normal samples and identified 22 functionally enriched DEGs. Moreover, we used two machine learning algorithms for the first time, to further screen possible biomarkers of CAVS, identifying *SCG2*, *PPBP*, *TREM1*, *CCL19*, *WIF1*, and *MMP9* as suitable candidates. Mitochondria, known as the “powerhouses” in cells, play essential roles in many cellular activities, including cell growth and death, signal transduction, and energy metabolism. An increasing number of studies have reported the important role of mitochondria in VHD progression. Interestingly, we identified a mitochondria-related gene, *MMP9*, as one of the mitochondrial dysfunction biomarkers for CAVS. Using the GSE83453 dataset, we further demonstrated that *MMP9* expression was distinctly higher in CAVS samples, compared with that in normal samples. In addition, ROC curve analysis revealed *MMP9* as a potential indicator to distinguish CAVS samples from normal samples, with an AUC of 0.921, highlighting its potential use as a novel diagnostic biomarker.

A thorough understanding of disease pathophysiology and basic science is required for drug development. Myofibroblast activation, osteoblastic transition, lipoprotein deposition, and inflammation play important roles in the pathogenesis of CAVS, and accordingly, lymphocytic infiltration is a defining feature thereof. However, most pharmaceutical strategies are absorbed in general cardiovascular health with focus on treatments for dyslipidemia, diabetes, and hypertension [21]. The enrichment analysis conducted herein indicated that the “IL-17 signaling pathway,” “ECM-receptor interaction,” “viral protein interaction with cytokine and cytokine receptor,” “chemokine signaling pathway,” and “focal adhesion” were noticeably enriched; accordingly, we were curious whether immune cell infiltration played a part in the pathogenic role of *MMP9* in CAVS. We found that *MMP9* expression was positively correlated with “macrophage M0,” “dendritic cells activated,” and “macrophage M2” confirming our postulation.

Finally, to demonstrate the results from online datasets, we performed western blotting and immunohistochemistry, which also confirmed that *MMP9* expression was distinctly increased in CAVS samples, compared to normal samples. Matrix metalloproteinases (MMPs)—a class of approximately 25 zinc-dependent proteinases—are involved in the regulation of several cellular functions, including angiogenesis [22], differentiation, proliferation, and apoptosis [23]. Of these, *MMP9* is reportedly involved in mitochondrial damage, which, in turn, has been confirmed to play an important role in the progression of CAVS. In this study, we found that the mitochondria of VICs were significantly fragmented, confirming the presence of mitochondrial damage in calcified VICs. However, inhibiting *MMP9* significantly improved mitochondrial morphology, mitochondrial metabolism, and oxidative stress. In addition, the calcification of VICs decreased significantly, in a dose-dependent manner. Our findings highlighted the important role of *MMP9* in the progression of CAVS by inducing an imbalance in mitochondrial quality.

## 5. Conclusion

For the first time, six novel biomarkers (*SCG2*, *PPBP*, *TREM1*, *CCL19*, *WIF1*, and *MMP9*) for CAVS have been identified, based on machine learning algorithms; these may be important regulators of CAVS progression. *MMP9*, a mitochondria-related gene, has been correlated with M0 macrophages, activated dendritic cells, and M2 macrophages, and its inhibition may attenuate cardiovascular calcification by reducing mitochondrial damage. Our findings suggest *MMP9* as a novel mitochondrial dysfunction biomarker and therapeutic target for CAVS.

However, this study has some limitations. First, despite the fact that different datasets were collected to confirm the diagnostic value of *MMP9*, the study has a retrospective design, and additional clinical samples are required to confirm our findings. Second, the potential function of *MMP9* in the immune microenvironment was not demonstrated using either in vitro or in vivo experiment. Third, the molecular mechanisms involved in *MMP9*-mediated mitochondrial quality control need to be further investigated. These factors offer scope for future research.

## Figures and Tables

**Figure 1:** Identification of DEGs in CAVS, along with functional enrichment analysis. (a) Volcanic map of identified DEGs between non-CAVS and CAVS samples. (b) GO and (c) KEGG analyses of DEGs.

**Figure 2:** Identification of diagnostic genes using two machine learning algorithms. (a) The LASSO regression algorithm was applied to screen diagnostic biomarkers of CAVS. (b) A plot of biomarker selection using the SVM-RFE algorithm. (c) Six diagnostic genes were identified based on the previous two algorithms. (d) A Venn diagram demonstrating mitochondria-related gene, *MMP9*, as a novel biomarker of CAVS.

**Figure 3:** Validation of the expression and diagnostic values of *MMP9* in the GSE83453 dataset. (a) *MMP9* expression was distinctly higher in CAVS samples. (b, c) ROC assays of *MMP9* expression based on the GSE83453 and GSE12644 + GSE51472 datasets, respectively.

**Figure 4:** CIBERSORT analysis of infiltrating immune cells in non-CAVS and CAVS groups. (a) The distribution of 22 immune cells in the non-CAVS and CAVS groups, respectively, portrayed in a stacked bar chart. (b) Correlation matrix of immune cell proportions. Positive and negative correlations are shown in red and blue, respectively. (c) Violin plot highlighting the differences in immune cell infiltration, between the non-CAVS and CAVS groups.

**Figure 5:** Correlations between *MMP9* expression and immune cell infiltration in CAVS. (a) The correlation analysis. (b) The bubble chart.

**Figure 6:** *MMP9* was highly expressed in CAVS. (a) RT-PCR, (b) western blotting, and (c) immunohistochemistry were conducted to examine the expression of *MMP9* in non-CAVS and CAVS samples, respectively (bar = 50 *μ*m). (d) CT images confirmed an obvious calcified focus in CAVS samples, and TEM images showed mitochondria cristae damage in aortic valve tissues (bar = 500 nm). (a) *p* < 0.05 compared with non-CAVS group.

**Figure 7:** *MMP9* inhibition attenuated calcification via suppression of mitochondrial quality imbalance. (a) MitoTracker Red staining immunofluorescence reflected the mitochondrial morphology in VICs. Mitochondrial aspect ratio was quantified by ImageJ (bar = 25 *μ*m). (b) FITC-ROS staining immunofluorescence reflected the oxidative stress in VICs (bar = 50 *μ*m). (c) The fluorescence intensity of DHE reflected the oxidative stress in VICs. (d) JC-1 aggregate/monomer ratio reflected the mitochondrial membrane potential in VICs (bar = 25 *μ*m). (e) Citrate synthase activity was detected to observe the mitochondrial metabolism in VICs. (f) Representative Alizarin Red stain and quantification of calcified VICs, treated with either MMP-9i (100 nM) or MMP-9i (300 nM). CM: control medium, OM: osteogenic medium. (a) *p* < 0.05 compared with CM-VIC group, (b) *p* < 0.05 compared with OM-VIC group, (c) *p* < 0.05 compared with the OM-VIC+ MMP-9i (100 nM) group.

## Data Availability

The datasets used and/or analyzed during the current study are available from the corresponding authors upon reasonable request.

## Supplementary Materials

Supplementary 1 Western blotting result showing the inhibitory effect of MMP-9i to the expression of MMP-9 (*n* = 3 samples/group). CM: control medium, OM: osteogenic medium. (a) *p* < 0.05 compared with CM-VIC group, (b) *p* < 0.05 compared with OM-VIC group, (c) *p* < 0.05 compared with the OM-VIC+ MMP-9i (100 nM) group.

Supplementary 2 The detailed images of FITC-ROS staining in VICs and quantification to Figure 7(b) (bar = 50 *μ*m). CM: control medium, OM: osteogenic medium. (a) *p* < 0.05 compared with CM-VIC group, (b) *p* < 0.05 compared with OM-VIC group, (c) *p* < 0.05 compared with OM-VIC+ MMP-9i (100 nM) group.

Supplementary 3 The detailed images of mitochondrial membrane potential and quantification to Figure 7(d) (bar = 25 *μ*m). CM: control medium, OM: osteogenic medium. (a) *p* < 0.05 compared with CM-VIC group, (b) *p* < 0.05 compared with OM-VIC group, (c) *p* < 0.05 compared with the OM-VIC+ MMP-9i (100 nM) group.
